RETRACTED

# Association of *MDR1* Gene SNPs and Haplotypes with the Tacrolimus Dose Requirements in Han Chinese Liver Transplant Recipients

**DOI:** 10.1371/journal.pone.0025933

**Published:** 2011-11-14

**Authors:** Xiaobo Yu, Haiyang Xie, Bajin Wei, Min Zhang, Weilin Wang, Jian Wu, Sheng Yan, Shusen Zheng, Lin Zhou

**Affiliations:** 1 Key Lab of Combined Multi-Organ Transplantation, The First Affiliated Hospital, School of Medicine, Zhejiang University, Ministry of Public Health, Hangzhou, Zhejiang, China; 2 Department of Surgery, Division of Hepatobiliary and Pancreatic Surgery, The First Affiliated Hospital, School of Medicine, Zhejiang University, Hangzhou, Zhejiang, China; University of California Los Angeles, United States of America

## Abstract

**Background:**

This work seeks to evaluate the association between the C/D ratios (plasma concentration of tacrolimus divided by daily dose of tacrolimus per body weight) of tacrolimus and the haplotypes of *MDR1* gene combined by C1236T (rs1128503), G2677A/T (rs2032582) and C3435T (rs1045642), and to further determine the functional significance of haplotypes in the clinical pharmacokinetics of oral tacrolimus in Han Chinese liver transplant recipients.

**Methodology/Principal Findings:**

The tacrolimus blood concentrations were continuously recorded for one month after initial administration, and the peripheral blood DNA from a total of 62 liver transplant recipients was extracted. Genotyping of C1236T, G2677A/T and C3435T was performed, and SNP frequency, Hardy-Weinberg equilibrium, linkage disequilibrium, haplotypes analysis and multiple testing were achieved by software PLINK. C/D ratios of different SNP groups or haplotype groups were compared, with a *p* value<0.05 considered statistically significant. Linkage studies revealed that C1236T, G2677A/T and C3435T are genetically associated with each other. Patients carrying T-T haplotype combined by C1236T and G2677A/T, and an additional T/T homozygote at either position would require higher dose of tacrolimus. Tacrolimus C/D ratios of liver transplant recipients varied significantly among different haplotype groups of *MDR1* gene.

**Conclusions:**

Our studies suggest that the genetic polymorphism could be used as a valuable molecular marker for the prediction of tacrolimus C/D ratios of liver transplant recipients.

## Introduction

To lower the risk of rejection after allogenetic organ transplantation, immunosuppressive drugs are widely used to reduce the immune system activity. Tacrolimus, also named FK506, is a kind of immunosuppressive drugs, and able to inhibit the multiplication of T-cells [1]. Postoperative patients have to take tacrolimus all their lives to make a better graft survival, which results in heavy financial costs [1]. The optimal use of tacrolimus could not only lower the financial cost but also reduce the side effects caused by tacrolimus, which makes it a valuable therapy for liver transplant recipients. However, pharmacokinetic characteristics of tacrolimus vary dramatically among individuals. Pharmacokinetic characteristics could be influenced in many ways, one of which may be the genetic factors including single nucleotide polymorphism (SNP), haplotype and DNA methylation [2], [3], [4], [5], [6].

RETRACTED

Human multidrug resistance (*MDR1*) gene, also named P-glycoprotein, is a member of the ATP-binding cassette superfamily. MDR1 protein anchors in cell membrane, and acts as an efflux transporter of various substrates for cell protection [4], [6]. It has been reported in the literature that tacrolimus is one substrate of MDR1 [5], [7], [8]. *MDR1* is polymorphic, and at least 50 SNPs have been found so far [4], [9], [10], [11], [12], [13]. The functional consequences of reported SNPs are not completely understood and still controversial to date. SNPs occur as a result of single-nucleotide substitutions in coding region and non-coding region, which might influence mRNA expression [14] and protein translation and folding [6], [8], and finally affect drug pharmacokinetic characteristics. Moreover, the allelic frequency of *MDR1* SNPs varies widely among ethnic groups [4], [5], [6]. Haplotype is a set of genetically associated SNPs [15], [16], [17], and can be mathematically calculated by software including PLINK and Haploview [18], [19]. Linkage studies showed that there is strong linkage disequilibrium among the highly frequent polymorphisms C1236T (rs1128503), G2677A/T (rs2032582) and C3435T (rs1045642) [6], [20], [21]. Furthermore, the effects of haplotype on drug response and disease outcome have been reported [20], [21], [22], [23]. Other studies on specific mechanism have demonstrated that haplotypes may alter mRNA stability [24], protein conformation and inhibitor efficiency [6].

Dose-adjusted trough concentration (concentration/dose [C/D], plasma concentration of drug divided by daily dose of drug per body weight) was used as the criteria for comparison among different SNP or haplotype groups in most of the previous studies [25], [26], [27], [28], [29]. We have already observed lower tacrolimus C/D ratios in liver transplant recipients of *MDR1* C3435T C/C homozygotes previously [28]. Our new findings not only supported the previous observation, but also provided the evidence that *MDR1* haplotype could affect tacrolimus C/D ratios.

## Methods

### Patients

The population in this study was Han Chinese, including 5 female and 57 male, aged from 21 to 64 years old (46.6±9.3), and weighed from 50 to 85 kg (66.4±8.4). For all the patients, tacrolimus-based immunosuppressive regimens were included. The oral administration of tacrolimus and steroid was introduced in our previous study [28].

RETRACTED

### Ethics statement

The research protocol was approved by the Institutional Review Board, Key Lab of Combined Multi-organ Transplantation, Ministry of Public Health. Informed written consent was obtained according to the Declaration of Helsinki.

### Data Collection and Therapeutic Drug Monitoring

After the initial administration of tacrolimus, all patients received clinical evaluations and laboratory tests in the first month. The daily dose (mg) of tacrolimus was recorded, and the weight-adjusted dosage (mg/kg/d) was calculated. Drug blood levels were measured by immunoassay on the IMx analyzer (Abbott Diagnostics Laboratories, Abbott-Park, IL). Dose-adjusted trough concentrations were calculated by dividing tacrolimus trough concentrations by the corresponding dose on an mg/kg basis (concentration/dose [C/D] ratio).

### Genotyping

Genomic DNA of patients was extracted from peripheral blood using QIAamp DNA Blood mini kit (QIAGEN, Hilden, Germany) following the manufacturer's instruction. RFLP (restriction fragment length polymorphism) PCR method was used to genotype the position C1236T, G2677A/T and C3435T. Primer pairs 5′ TTCACTTCAGTTACCCATC 3′ and 5′ CATAGAGCCTCTGCATCA 3′ and restriction enzyme *Bsu*RI were used to distinguish T allele from C allele of C1236T, with primer pairs 5′ AGAGCATAGTAAGCAGTAGGGAGTA 3′ and 5′ GCAAATCTTGGGACAGGAATA 3′ and restriction enzyme *Rsa*I for distinguishing A allele from G or T allele of G2677A/T, primer pairs 5′ AGTAAGCAGTAGGGAGTAACA 3′ and 5′ GATAAGAAAGAACTAGAACGT 3′ and restriction enzyme *Acl*I for distinguishing T allele from G or A allele of G2677A/T, primer pairs 5′ GATCTGTGAACTCTTGTTTTCA 3′ and 5′ GAAGAGAGACTTACATTAGGC 3′ and restriction enzyme *Mbo*I for distinguishing T allele from C allele of C3435T. PCR and products digestion by restriction enzyme were performed as reported [30].

### Statistical Analysis

Nonparametric tests, including Mann-Whitney test and Kruskal-Wallis test, were applied to assess significance test for comparisons of all group pairs, with a further confirmation by multiple test, max(T) permutation by 10000 times. Nonparametric tests were performed by Graphpad Prism 5.03 (Graphpad Software, San Diego, CA, USA). Hardy-Weinberg equilibrium, linkage disequilibrium, haplotype frequency analyses and max(T) permutation were performed by PLINK v1.06 (http://pngu.mgh.harvard.edu/purcell/plink/). The expectation-maximization (E-M) algorithm was used to estimate haplotype frequencies by PLINK. A *p* value<0.05 was considered statistically significant.

RETRACTED

## Results

### Genotype Frequency of patients

All single SNP genotypes were recorded, and frequencies were calculated. No statistical significance was found among genotype groups related to gender, age and weight (Table 1). Results of Kruskal-Wallis tests were not shown. As mentioned in *method*, PLINK was used to analyze Hardy-Weinberg equilibrium, linkage disequilibrium and haplotype frequencies. G2677A/T has 3 alleles, however, according to the user manual, PLINK is unable to analyze SNPs with more than 2 alleles. Therefore, when one allele was compared with other two alleles, there had to be a new character to represent the two alleles. In accordance to the IUPAC (Union of Pure and Applied Chemistry) coding standards, ‘K’ was used as the abbreviation for T and G alleles, with ‘R’ for A and G alleles together and ‘W’ for A and T alleles together. So G2677A/T was also named as G2677A/T(A-K), G2677A/T(T-R) or G2677A/T(G-W). All three SNPs frequencies were in accordance with Hardy-Weinberg equilibrium, and the *p* value were >0.05 (Table 2).

**Table 1:** Demographic characteristics of liver transplant patients.

SNP	Genotype	*N*	Gender(M/F)	Age (mean ± S.D.)	Weight, kg (mean ± S.D.)
C1236T	C/C	9 (14.5%)	9/0	47.9±9.5	69.3±8.4
	C/T	25 (40.3%)	24/1	44.8±9.4	68.7±8.5
	T/T	28 (45.1%)	24/4	47.9±9.1	63.4±7.5
G2677A/T	A/A	2 (3.2%)	2/0	43.0±11.3	65.5±9.2
	A/G	8 (12.9%)	8/0	49.6±6.5	71.1±7.7
	A/T	6 (9.7%)	5/1	40.0±12.5	69.2±9.6
	G/G	16 (25.8%)	15/1	48.4±6.4	63.1±8.7
	G/T	22 (35.4%)	20/2	46.8±10.8	67.0±7.9
	T/T	8 (12.9%)	7/1	45.4±8.8	62.1±7.0
C3435T	C/C	7 (11.3%)	6/1	46.6±8.8	60.7±6.2
	C/T	24 (38.7%)	24/1	44.8±10.8	66.3±8.0
	T/T	31 (50%)	28/3	48.0±8.0	67.7±8.7

**Table 2:** SNPs frequencies in liver transplant patients.

SNP position	Alleles Frequency		Genotypes Frequency		Hardy–Weinberg equilibrium			Comparison of C/D ratios	
	Allele	N	Genotype	N	O(HET)^d^	E(HET)^e^	*p*	C/D ratios	*p*
C1236T	C	43 (34.7%)	C/C	9 (14.5%)	0.4032	0.453	0.4048	143.50±37.99	0.6772
	T	81 (65.3%)	C/T	25 (40.3%)				142.73±39.23	
			T/T	28 (45.1%)				138.26±47.61	
G2677A/T(A-K)^a^	A	18 (14.5%)	A/A	2 (3.2%)	0.2258	0.2482	0.5985	146.20±35.66	0.4166
	K	106 (85.5%)	A/K	14 (22.6%)				139.01±44.86	
			K/K	46 (74.2%)				152.23±50.23	
G2677A/T(T-R)^b^	T	44 (35.5%)	T/T	8 (12.9%)	0.4516	0.4579	1	145.35±41.76	0.2677
	R	80 (64.5%)	T/R	28 (45.2%)				141.73±44.17	
			R/R	26 (41.9%)				122.77±38.51	
G2677A/T(G-W)^c^	G	62 (50.0%)	G/G	16 (25.8%)	0.4839	0.5	0.8025	148.33±45.48	0.5398
	W	62 (50.0%)	G/W	30 (48.4%)				137.76±42.17	
			W/W	16 (25.8%)				138.82±41.98	
C3435T	C	38 (30.6%)	C/C	7 (11.3%)	0.3871	0.4251	0.5496	117.54±23.16	0.0419
	T	86 (69.4%)	C/T	24 (38.7%)				137.95±49.83	
			T/T	31 (50%)				150.20±48.05	
			C/C					117.54±23.16	0.0240
			C/T+T/T					144.20±40.05	

a the character ‘K’ is for T, thymine, or G, guanine.

b the character ‘R’ is for A, adenine, or G, guanine.

c the character ‘W’ is for A, adenine, or T, thymine.

d O(HET) is short for observed heterozygosity.

e E(HET) is short for expected heterozygosity.

RETRACTED

### Effect of SNPs on Tacrolimus Dose Requirement

Data of oral tacrolimus dose was collected, and the relationship between *MDR1* SNP genotypes and C/D ratio was investigated. No statistically significant association was observed in position C1236T and G2677A/T, except C3435T (Table 2). Similar to the results of our previous study [28], we found that recipients with C/C genotype at C3435T would require a little higher dose of tacrolimus compared to those with C/T and T/T genotypes (Table 2).

It was reported that linkage disequilibrium existed in C1236T, G2677A/T and C3435T, and association among the three SNPs, also called haplotype, might influence drug pharmacokinetics. So we tested the linkage disequilibrium of all pairs of these three SNPs at the beginning. When C1236T combined with C3435T, or G2677A/T combined with C3435T, linkage disequilibrium was found (Table 3). C1236T also had linkage disequilibrium with G2677A/T(A-K) and G2677A/T(T-R), not with G2677A/T(G-W) (Table 3). And then according to the result of linkage disequilibrium, haplotype frequency analyses were performed, which do not include the combination between C1236T and G2677A/T(G-W). The haplotypes of individuals were recorded. No statistical significance was found in either of the 6 different pairs of combination (Table 4). But when C1236T and G2677A/T(T-R) were combined, patients with T-T/T-T, T-T/C-T and T-T/T-R haplotypes showed lower C/D ratios than those with T-R/T-R, T-R/C-R, T-T/C-R and C-R/C-R, which meant that patients carrying T-T haplotype and with an additional T/T homozygote at position C1236T or G2677A/T would require higher dose of tacrolimus (Table 5). Furthermore, it seemed that patients with T-C/T-C or T-C/R-T haplotypes showed lower C/D ratios than those with other haplotypes, which meant patients carrying T-C haplotype with the combination of G2677A/T(T-R) and C3435T required higher dose of tacrolimus to maintain serum concentration. However, after the max(T) permutation adjustment, no statistical significance was observed (Table 5).

**Table 3:** Haplotype analysis of different pairs of the three SNPs.

Combined SNPs	Haplotypes	*N*	LD^a^
C1236T vs G2677A/T(A-K)	C-A	17 (13.5%)	D′ = 0.897
	T-A	1 (1%)	
	C-K	26 (21.1%)	
	T-K	80 (64.3%)	
C1236T vs G2677A/T(T-R)	C-T	4 (3.4%)	D′ = 0.724
	T-T	40 (32.1%)	
	C-R	39 (31.3%)	
	T-R	41 (33.2%)	
C1236T vs G2677A/T(G-W)	C-W	21 (17.3%)	D′ = 0.000
	T-W	41 (32.7%)	
	C-G	21 (17.3%)	
	T-G	41 (32.7%)	
C1236T vs C3435T	C-C	1 (1.1%)	D′ = 0.895
	T-C	37 (29.5%)	
	C-T	42 (33.6%)	
	T-T	44 (35.8%)	
G2677A/T(A-K) vs C3435T	A-C	0 (0%)	D′ = 1.000
	K-C	38 (30.6%)	
	A-T	18 (14.5%)	
	K-T	68 (54.8%)	
G2677A/T(T-R) vs C3435T	T-C	35 (28%)	D′ = 0.868
	R-C	3 (2.6%)	
	T-T	9 (7.4%)	
	R-T	77 (61.9%)	
G2677A/T(G-W) vs C3435T	W-C	34 (27.5%)	D′ = 0.796
	G-C	4 (3.1%)	
	W-T	28 (22.5%)	
	G-T	58 (46.9%)	

a LD, linkage disequilibrium.

RETRACTED

**Table 4:** Tacrolimus concentration/dose (C/D) ratios of different haplotype groups.

Combined SNPs	Haplotypes	*N*	C/D	Combined SNPs	Haplotypes	*N*	C/D
C1236T - G2677A/T(A-K)	C-A/C-A	1 (1.6%)	188.07±0.00	G2677A/T(A-K) - C3435T	A-T/A-T	2 (3.2%)	156.40±43.84
	C-A/T-K	9 (14.5%)	147.86±44.63		A-T/K-C	4 (6.5%)	149.08±29.46
	C-K/C-A	5 (8.1%)	128.09±40.17		K-T/A-T	10 (16.1%)	142.79±35.38
	C-K/C-K	3 (4.8%)	116.71±40.46		K-T/K-T	19 (30.6%)	137.01±41.89
	T-A/C-A	1 (1.6%)	177.61±0.00		K-T/K-C	20 (32.3%)	145.33±49.36
	T-K/C-K	15 (24.2%)	145.89±47.77		K-C/K-C	7 (11.3%)	126.42±38.70
	T-K/T-K	28 (45.2%)	137.47±39.28				
C1236T - G2677AT-(T-R)	C-R/C-R	8 (12.9%)	135.65±41.19	G2677AT-(T-R) - C3435T	R-T/R-T	23 (37.1%)	139.23±36.19
	C-R/C-T	1 (1.6%)	93.44±0.00		R-T/R-C	3 (4.8%)	192.31±46.51
	C-R/T-T	12 (19.4%)	146.65±41.54		R-T/T-T	7 (11.3%)	149.24±49.34
	T-R/C-R	11 (17.7%)	141.91±44.64		T-T/T-T	1 (1.6%)	97.17±0.00
	T-R/T-R	7 (11.3%)	142.06±30.32		T-C/R-T	21 (33.9%)	139.10±42.89
	T-R/T-T	15 (24.2%)	135.15±38.28		T-C/T-C	7 (11.3%)	126.42±38.70
	T-T/C-T	2 (3.2%)	188.07±62.59				
	T-T/T-T	6 (9.7%)	138.83±53.93				
C1236T - C3435T	C-T/C-T	9 (14.5%)	130.97±42.39	G2677A/T(G-W) - C3435T	G-T/G-T	13 (21.0%)	138.18±37.49
	C-T/T-C	10 (16.1%)	147.61±44.29		G-T/G-C	3 (4.8%)	192.31±46.51
	T-T/C-T	14 (22.6%)	148.35±49.13		G-T/W-T	13 (21.0%)	138.66±40.31
	T-T/T-T	8 (12.9%)	137.06±36.82		W-T/W-T	5 (8.1%)	149.00±49.54
	T-T/T-C	14 (22.6%)	137.15±36.54		W-T/W-C	4 (6.5%)	149.08±29.46
	T-C/C-C	1 (1.6%)	143.82±0.00		W-C/G-T	17 (27.4%)	137.04±44.43
	T-C/T-C	6 (9.7%)	138.83±43.93		W-C/W-C	7 (11.3%)	126.42±38.70

**Table 5:** Statistical analysis of tacrolimus concentration/dose (C/D) ratios at 1 month after drug initiation between haplotype groups.

SNP position	Haplotypes	C/D	*p*
C1236T - G2677A/T(A-K)	T-T/T-T+T-T/C-T+T-T/T-R	128.65±43.60	0.0156
	T-R/T-R+T-R/C-R+T-T/C-R+C-R/C-R	148.14±40.40	0.034#
G2677A/T(T-R) - C3435T	T-C/T-C+T-C/R-T	132.45±37.16	0.049
	R-T/R-T+R-T/R-C+R-T/T-T	151.85±39.23	0.098#

# indicated the *p* value given by max(T) permutation.

## Discussion

It has been reported that there are more than 50 SNPs in human *MDR1* gene [9], [10], [11], [12], [13], [31]. SNPs spread from the 5′ start to the 3′ untranslated region in *MDR1* transcript, resulting in both synonymous and non-synonymous mutations [4], [5], [6]. Three SNPs, C1236T, G2677A/T and C3435T, all locate in exons. Mutation of G2677A/T causes coding sequence missense, while the others are synonymous [5]. Missense substitutions in amino acid may result in abnormal protein folding, moreover, there has been a hypothesis that the presence of rare codons, marked by synonymous polymorphisms, may affect the insertion of MDR1 into the membrane and alter the structure of substrate interaction sites [8]. These SNPs have become research focus, which include effects of SNPs and haplotypes in different ethnic groups [7], [13], [32], [33], [34], [35], [36], [37], [38] on *MDR1* mRNA stabilization [24], [39], [40], [41] or protein expression and folding [5], [10] in patients, and effects on substrates efflux in cell models [5], [8].

RETRACTED

According to the literature mentioned above, both G2677A/T and C3435T have significant association with tacrolimus or cyclosporine pharmacokinetics, and their clinical behaviors exhibit significantly different requirements of drug dose among different SNP groups. Recipients with C/C homozygotes of *MDR1* in position C3435T showed significantly lower dose-adjusted tacrolimus concentrations compared with the other groups [28], [37], [42]. Since the ethnic population was Han Chinese, the same population in our previous study [28], similar phenomenon was observed. Some other research groups also identified SNPs related to cyclosporine pharmacokinetics, still there are controversies. In some cases, recipients with C/C homozygote in position C3435T required higher dose of cyclosporine [43], [44], while others did not [45], [46], [47]. One of the explanations is that SNPs frequencies may vary quite differently depending on specific ethnic groups, for instance, homozygosity for T allele in position C1236T is 37.5%in Japanese [48], while 13.3% in Caucasians [11]. Different ethnic populations have different SNP frequencies at the same position, which may cause the controversial results.

Genetic association of SNPs, named haplotypes [15], [16], was also found to influence drug pharmacokinetics on *MDR1* genotype-phenotype correlation in further studies [6], [20], [49]. Haplotypes analysis in this work provided the evidence that genetic association existed between each other among C1236T, G2677A/T and C3435T, and haplotypes of *MDR1* influenced tacrolimus concentration/dose (C/D) ratios in liver transplant recipients. Our findings showed that recipients who carried T-T haplotype and an additional T/T homozygote at either SNPs required higher doses, when C1236T and G2677A/T were combined. The association between haplotypes for G2677A/T and C3435T and tacrolimus C/D ratio was weak after max(T) permutation adjustment.

RETRACTED

Patients who have received a new liver, with a different genetic background, will metabolize drugs in different ways. Dose requirements of tacrolimus would be predicted much more precisely, if genetic polymorphism of *MDR1* is investigated both in donors and recipients. And several research groups have obtained some helpful results [25], [28], [50].

The ultimate goal of human genetics and genomics studies is to understand the mechanism of gene interaction networks, which would finally explain how gene-drug interactions work [51]. Based on these efforts, pharmacologists and physicians hope that the individualized drug therapy would become reality one day. It is not difficult to identify genes contributing to some phenotype, such as drug pharmacokinetics. However, the phenotype is seldom monogenic. Lots of genes, including downstream molecules, are implicated in biological regulation. To facilitate the identification of these genes, new genome-wide research techniques have been developed. The Affymetrix or Illumina SNP chips are the newest human GWAS (genome wide association study) methods, which produce high throughput SNP data from big ethnic populations with high costs. For instance, by analyzing Affymetrix SNP chips data of a population suffering SLE (systemic lupus erythematosus), several susceptibility genes participating in network of immune response and signal regulation pathway were identified, including immune complex processing and immune signal transduction in lymphocytes [52]. However, only large research groups with enough budgets could afford it. For most research groups, it would be quite sensible to pick up some candidates from databases, and investigate in replicate populations followed by mechanism studies. For those SNPs, which have been proved clinically effective, genotyping with a cost of less than 1 US dollar for each site could significantly promote the development of individualized drug treatment.

In conclusion, our results provided new evidence of the association of *MDR1* and tacrolimus dose requirements, which could be a great help to the individualized tacrolimus treatment of liver transplant recipients.
